# Loneliness Status and Related Factors among the Hakka Elderly in Fujian, China: Based on the Health Ecological Model

**DOI:** 10.1155/2022/2633297

**Published:** 2022-08-21

**Authors:** Huajing Chang, Yimin Huang, Xiaojun Liu

**Affiliations:** ^1^Department of Health Management, School of Public Health, Fujian Medical University, Fuzhou, Fujian 350122, China; ^2^Hunan Provincial Key Laboratory of Clinical Epidemiology, Xiangya School of Public Health, Central South University, Changsha, Hunan 410078, China

## Abstract

There are few studies estimating the loneliness of the Hakka elderly in China. This study aims to examine the loneliness status and related factors among the Hakka elderly in Fujian, China. The short-form UCLA Loneliness Scale (ULS-8) was used to assess the loneliness of the Hakka elderly. Factors associated with loneliness were classified as individual indicators, behavioral indicators, interpersonal indicators, and social indicators according to the health ecological model (HEM). Hierarchical linear regression models were established to identify the main factors that were most predictive of loneliness. A sample of 1,262 Hakka elderly people was included in this study. Females (*β* = 0.631, *P*=0.012), those with ≥2 chronic diseases (*β* = 1.340, *P* < 0.001), those who were currently living in rural areas (*β* = 4.863, *P* < 0.001) or suburban areas (*β* = 2.027, *P* < 0.001), those with parents both died (*β* = 0.886, *P*=0.001), and those with the Urban Employees Basic Medical Insurance (UEBMI; *β* = 0.852, *P*=0.030) obtained a higher score of ULS-8. Those exercised regularly (*β* = −2.494, *P* < 0.001), those had leisure activities (*β* = −1.937, *P* < 0.001), those ate healthy (*β* = −1.270, *P* < 0.001), and those with better self-rated financial status and higher education level received a lower score of ULS-8. There are differences in loneliness among different Hakka elderly population subgroups, and healthy behaviors and lifestyles may reduce the loneliness of the Hakka elderly. Relevant interventions should be implemented in a targeted manner, focusing on susceptible populations. This is most evident among those who were female, living in rural areas, with parents both died, with lower education, and with multiple chronic diseases.

## 1. Introduction

As the medical model shifted to the biopsychosocial medical model, issues related to mental health are receiving increasing attention, most notably loneliness. Loneliness is a unique psychological feeling, which has an important impact on human health [1]. Loneliness is usually defined as a painful feeling of social isolation [2], which is a subjective and negative feeling due to the individual's perception of a lack of social interaction or poor social relationships [3–5]. Globally, the prevalence of loneliness ranged from 10.5% to 34% [6–8]. A meta-analysis showed that the pooled prevalence estimate of loneliness was 28.5% [9]. Loneliness may occur in any age group, and it is believed to be a common and more serious problem for older adults [10]. With ageing, the physical function of older adults gradually declines and the number of chronic diseases increases, combined with retirement and the death of a spouse or significant other, loneliness is more prevalent in older adults [11,12]. Some research showed that loneliness could lead to ill health [13], poor prognosis [14], and impaired quality of life [15] with cognitive decline, depression, stress, and anxiety [16–19]. It is even associated with an increased risk of suicide and mortality [20,21].

The global population is ageing rapidly. By 2050, the world's population aged 60 years and older is expected to total 2 billion [22]. Loneliness among older people has become a serious global public health issue. In high-income countries, loneliness is common among older adults affecting approximately one in four [9]. As the largest developing country with the largest elderly population, China needs to attach more importance to loneliness. Especially in the context of rapid social changes, some special problems among the elderly have arisen, including a rising number of empty-nest and left-behind older adults. Consequently, the prevalence of loneliness among the elderly in China is getting higher than before and also likely to be higher than that in other countries [23]. A large proportion of current research on loneliness have been conducted in developed countries, while studies about loneliness among the elderly in Chinese populations are comparatively sparse. A study on the elderly in Shanghai showed that the old-old had a higher level of loneliness than the young-old [24]. There were 58.1% of older people in Hong Kong reported a high level of loneliness [1], and the prevalence of loneliness among older adults in Taiwan was 10.5% [25]. Given the increasing prevalence of loneliness in the elderly and the undesirable consequences of loneliness, it is imperative to pay more attention to the loneliness of the elderly and its related factors in China.

Numerous fragmented studies have shown that loneliness was associated with gender, age, marital status, living arrangement, education level, family income, health-related behaviors, health status, and so on [1,5,6,8,11,24,25]. Some research also discovered that loneliness is associated with culture and nationality [26,27]. An individual's cultural background could affect that person's experience of loneliness. The elderly in more collectivist societies tend to be more lonely than those in individualistic countries [28]. Owing to the collective culture of the Chinese, older people may experience more loneliness due to reduced interactions with family members, as most young couples opt to form a nuclear family [1]. Besides, people may be reluctant to acknowledge loneliness because of the Chinese cultural influence. Chinese people, especially the elderly who hold traditional ideas and cultural beliefs, often have the feeling of social stigma and are more ashamed to express their true inner thoughts and feelings, which could lead to an underestimated prevalence of loneliness among the elderly in China. China is a multiethnic and multicultural country with 56 ethnic groups. Han, as the most populous ethnic group, accounts for 91.11% of the total population of China and has many internal branches [29]. The Hakka is a branch of the Han ethnic group and one of the far-reaching subnations that have a wide distribution in the history of China [30]. There are about 80 million Hakkas in the world, and about 50 million are distributed in Guangdong, Jiangxi, and Fujian of China, which is much larger than the Zhuang ethnic group, the most populous of the minority groups with 19.57 million clansmen [31]. Compared with the general elderly, the Hakka elderly's unique demographic characteristics and lifestyles may influence the level of loneliness.

However, there is limited study addressing the loneliness of the Hakka elderly. Therefore, this study aims to explore the loneliness status of the Hakka elderly in Fujian and to identify its potential correlates based on the health ecology model (HEM). The HEM includes individual indicators, behavioral indicators, interpersonal indicators, social indicators, and so on [32]. The present study is designed to obtain useful baseline information for the local, regional, and even national governments in China in their attempts to develop more effective health-prevention programs and strategies for reducing the level of loneliness in the Hakka elderly. Moreover, the findings of this study will become a starting point to draw the public's attention to the health conditions of the Hakka elderly and bridge the gap between scientific research and public awareness of the loneliness of the Hakka elderly.

## 2. Materials and Methods

### 2.1. Study Design and Participants

Data collection for the present study was nested in a larger cross-sectional population-based survey named China's Health-Related Quality of Life Survey for Older Adults 2018 (CHRQLS-OA 2018) [33]. The survey was organized and conducted by the Global Health Institute of Wuhan University during the Spring Festival in 2018, aiming to collect data on the socioecological factors and health status of the elderly. The samples from Ninghua, Fujian, which is commonly known as the cradle of the Hakka, were selected from the general database of the CHRQLS-OA 2018. Our study subjects were residents aged 60 years or older, had a local household registration, and voluntarily participated in the survey. However, those who had critical illnesses such as aphasia, deafness, blindness, paraplegia, and so on; had severe mental disorders; had been diagnosed with dementia; or had a history of mental illness were excluded from the survey. Considering the low education level of the elderly aged 60 or above in China, a face-to-face interview style was adopted in this study. For those with poor reading and response abilities, we asked their family caregivers for help. We distributed a total of 1,500 paper questionnaires, but some potential participants refused to participate in the study at the very beginning, and some quit during the interview. Hence, the present study only included 1,262 valid samples in the final analysis with a valid survey response rate of 84.13%.

### 2.2. Measures

In this study, the individual variables of the participants were divided into four layers according to the HEM: (1) individual layer was measured by four indicators: sex, age, self-rated health status, and number of NCDs. Age was grouped into five categories, namely, 60–64, 65–69, 70–74, 75–79, and ≥80. (2) Behavioral layer included five health-related behavioral indicators: regular exercise, leisure activities, healthy diet, smoking, and drinking. The standard of regular exercise was determined in accordance with the Chinese Center for Disease Control and Prevention (CDC), that is, participants who do exercise more than 3 times per week and at least 30 minutes per time were identified as regular exercise. Individuals who self-reported having self-determined activities (such as playing cards, Mahjong, chess, etc.) that happened outside of obligatory time were identified as having leisure activities. Individuals who self-reported having breakfast basically every day and having a balanced diet were considered to have healthy dietary behaviors. Participants who self-reported smoking at least one cigarette per week were defined as smokers, and who self-reported drinking more than one time per week were defined as drinkers. (3) Interpersonal layer involved four indicators: marital status, current residence, living arrangement, and survival of parents. Participants were divided into three subgroups based on their marital status, namely, married/cohabitation, widowed, and others (unmarried/divorced, separated, etc.). The living arrangement of participants included living alone, living with spouse only, living with children, mixed habitation, and others (only living with grandchildren/others/nursing home). (4) Social layer covered four indicators: working status, self-rated financial status, education level, and medical insurance. Education level fell into four groups, namely, illiterate, literacy class/home school, primary school, and junior high school and above (including vocational education). The theoretical framework is shown in Figure 1.

The present study employed the short-form UCLA Loneliness Scale (ULS-8) to assess the loneliness of the Hakka elderly. This scale was designed by Hays and Dimatteo; it consists of eight items selected from the revised UCLA Loneliness Scale [34,35]. The ULS-8 employs a four-point Likert scale for item scoring, and the response scale for questions estimating participants' rating of loneliness is 1 (never), 2 (seldom), 3 (sometimes), and 4 (always). Participants who had a higher total score were considered to have a higher level of loneliness. Among these eight items, there are two items that need to be reverse-coded. For the past few years, the ULS-8 was widely used for evaluating participants' loneliness, and many Chinese scholars have confirmed its reliability and validity of it [36,37]. Cronbach's alpha of the ULS-8 in this study is 0.947.

### 2.3. Statistical Analyses

Data analysis was performed in the following steps: first, an initial descriptive analysis was conducted. The frequencies and proportions were used to summarize the variables of each layer, and the means and standard deviations (SD) were used to calculate the score of loneliness. Then, *t*-tests and one-way analysis of variance (ANOVA) were applied to examine the statistical difference in ULS-8 scores. Lastly, we employed the hierarchical linear regression analysis to establish the regression models of loneliness and its related factors among the Hakka elderly. There were four models in this step. According to the HEM, we added variables associated with individual indicators in model 1. Model 2 added behavioral indicators on the basis of model 1. Models 3 and 4 added interpersonal indicators and social indicators, successively. The value of Durbin–Watson test statistic was close to 2.0, and the VIF values of all independent variables in the model are between 1.146 and 3.473 (all below 10). The Statistical Package for the Social Sciences (SPSS) version 23.0 for Windows (IBM Corporation, Armonk, NY, USA) was employed to conduct all statistical analysis work. The *P*-value of less than 5% was considered to be statistically significant.

### 2.4. Ethical Statement

The study was conducted according to the Declaration of Helsinki, and it had been approved by the Institutional Review Board of the School of Health Science and Faculty of Medical Sciences, Wuhan University (IRB number: 2019YF2050). Each questionnaire included informed consent information, which would be introduced before the surveys. Only those who were willing to voluntarily participate in and signed the informed consent form were considered our final respondents in the survey. The survey was also conducted anonymously, and the information of participants was kept confidential and only used for scientific research.

## 3. Results

### 3.1. Demographic Characteristics and the ULS-8 Scores of the Hakka Elderly

The final sample for this study included 1,262 Hakka elderly people, and their demographic characteristics were also demonstrated in our other published papers [38]. In this study, we found that the mean and standard deviation of the Hakka elderly's loneliness score was 16.27 ± 6.798. The results showed that there were statistically significant differences in ULS-8 scores among the indicators of sex (*t* = −5.363, *P* < 0.001), self-rated health status (*F* = 196.229, *P* < 0.001), number of NCDs (*F* = 55.497, *P* < 0.001), marital status (*F* = 125.117, *P* < 0.001), current residence (*F* = 558.301, *P* < 0.001), living arrangement (*F* = 80.191, *P* < 0.001), survival of parents (*t* = 8.228, *P* < 0.001), working status (*t* = −10.918, *P* < 0.001), self-rated financial status (*F* = 253.870, *P* < 0.001), education level (*F* = 224.965, *P* < 0.001), and type of medical insurance (*F* = 111.484, *P* < 0.001). Significantly lower ULS-8 score was observed in elderly individuals having regular exercise (*t* = 31.652, *P* < 0.001), leisure activities (*t* = 25.691, *P* < 0.001), and healthy diet (*t* = 15.559, *P* < 0.001). The details are shown in Table 1.

### 3.2. Hierarchical Linear Regression Analysis on the Loneliness Score of the Hakka Elderly

After checking the assumptions of hierarchical linear regression, we conducted this statistical analysis method according to the HEM. The loneliness score was taken as the dependent variable, and the 15 independent variables that detected differences in loneliness among the elderly in the last stage of the analysis were included in the model analysis. Model 1–4 added the variables of individual indicators, behavioral indicators, interpersonal indicators, and social indicators, successively. Model 4 is the final parsimonious model, and the results showed that females (*β* = 0.631, *P*=0.012), those with general (*β* = 0.819, *P*=0.004) or very poor/poor (*β* = 2.457, *P* < 0.001) self-rated health status, those with ≥2 chronic diseases (*β* = 1.340, *P* < 0.001), those who were widowed (*β* = 0.944, *P*=0.008), those who were currently living in rural areas (*β* = 4.863, *P* < 0.001) or suburban areas (*β* = 2.027, *P* < 0.001), those with parents both died (*β* = 0.886, *P*=0.001), those who still engaged in labor work (*β* = 1.128, *P* < 0.001), and those with the UEBMI (*β* = 0.852, *P* = 0.030) obtained a higher score of ULS-8, and those exercised regularly (*β* = −2.494, *P* < 0.001), those had leisure activities (*β* = -1.937, *P* < 0.001), those had healthy diet (*β* = −1.270, *P* < 0.001), those with general (*β* = −1.376, *P* < 0.001) or very good/good (*β* = −2.024, *P* < 0.001) self-rated financial status, and those with literacy class/home school (*β* = −1.527, *P* < 0.001) or primary school (*β* = −1.370, *P*=0.002) or junior high school or above (*β* = −2.105, *P* < 0.001) education level received a lower score of ULS-8. With the addition of variables at each layer, the fitting degree of the regression model was significantly improved, and the power of the model to explain the total variance continued to increase. Finally, model 4 explained 68.0% of the variance of the loneliness score. The details are shown in Table 2.

## 4. Discussion

The problem of loneliness in the Chinese elderly is unoptimistic. Previous studies showed that a number of Chinese older adults have moderate to severe levels of loneliness [2]. In this study, we found that the mean of the Hakka elderly's loneliness score was 16.27, which means the participants had moderate levels of loneliness and it is not very high as predicted. This would be attributed to the following possible reasons: (1) the survey population is relatively special; the Hakka people have their unique clan culture and folk belief. Some evidence indicated that religion could affect one's approach to life, behavior, and social involvement [39]. By participating in religious groups or denominations and attending religious services and related activities (such as prayer, meditation, etc.), the Hakka elderly can bolster their social networks and support, buffer against stressors, and improve their self-esteem and adaptive problem-solving ability, which could reduce the level of loneliness. (2) The overall health literacy level of the elderly in China is low, which is related to the low education level of the elderly in China [2]. Consistent with that, the Hakka elderly commonly have lower mental health literacy and cognition, and they may be reluctant to acknowledge the feeling of being lonely and believe that direct admission could be associated with compromising their self-worth [23]. (3) The survey was conducted during Chinese New Year, a time of year when family members were reunited annually. Accompanying by families and friends, the participants might underestimate their loneliness. (4) The subjects in this study were all from Ninghua, a place where the elderly population has relatively little mobility, or only intraprovincial mobility in the short term, which is bound to have little impact on the loneliness of the elderly caused by separation from relatives and friends. It is important to note that this study did not compare the status of loneliness level with other general populations (e.g., Han Chinese elderly population). Therefore, the differences between the loneliness of the Hakka elderly and the general population or other ethnic minority populations need to be further studied.

A range of indicators of demographic characteristics have been identified as potential predictors of loneliness, and some research reported that the loneliness of old people was relevant to sex, age, and physical health [40–42]. In this study, the male Hakka elderly reported a lower level of loneliness than females, which is consistent with other studies [43,44]. It may be because females are more willing to express their emotions, and males may be less likely to admit their feelings of loneliness, which produced some survey bias and the level of loneliness in males may be underestimated. Of course, it is also related to the sex differences in social roles and expectations. Women always play the role of housewives in China, which lead them to participate in fewer social activities and have more narrow social networks than men. An interesting finding of the present study was that there were no statistically significant differences in the level of loneliness among different age groups, which confirms that loneliness is common at all ages. What's more, we found that participants with poorer self-rated health status had higher loneliness scores. Compared with people without chronic diseases, people with chronic diseases had higher loneliness scores, and the more chronic diseases people had, the more lonely they felt, which reminds us that illness not only brings physical pain to people but also interacts with people's mental health. Therefore, it is suggested that more attention should be paid to the mental health of patients with chronic diseases and take measures to reduce their loneliness.

Health-related behavioral factors could reflect a person's psychological state. Related research showed that changes in loneliness were linked with changes in health-related behavior and living arrangement. Improvements in physical health were linked to reduced levels of loneliness [39]. This study found that those who exercised regularly, had leisure activities, ate healthily, and did not smoke received a lower score of ULS-8. These findings are in line with previous research [45,46]. However, the difference from previous studies is that we did not find that drinking was associated with loneliness among the Hakka elderly. There has been a distinct drinking culture in China spanning thousands of years, and alcohol consumption has an important place in many cultural celebrations. On the one hand, drinking is a social activity. Chinese people drink with others in order to build or maintain good interpersonal relationships, strengthen social ties, and broaden their social capital [47]. On the other hand, Chinese people believe they can “drink their sorrow away”; thus, they will drink alcohol to alleviate the feeling of loneliness. Some studies reported that moderate drinking can reduce loneliness, which is related to alcohol consumption [48]. Therefore, further research could attempt to investigate whether the amount of alcohol consumed is related to loneliness.

Social network size and composition had been widely recognized to be related to loneliness [49]. In this study, participants living in suburban areas had a higher level of loneliness than that living in urban areas but lower than that living in rural areas, which may be because there are more empty-nest elderly living in rural areas. With the rapid expansion of the Chinese economy, a growing number of young people left villages to seek employment elsewhere, leaving their parents as the empty-nest elderly to live by themselves. However, the social support systems for old people have not been well established, which caused the empty-nest elderly to have poorer physical and mental health [50]. Moreover, we found that the loneliness scores of the Hakka elderly living with children were relatively low, while the old people who lived alone or whose parents both died had higher scores. It showed that social support and frequent contact with family members were important in preventing and alleviating loneliness, which partially supports the traditional Chinese values of “the more children, the more happiness.” Loneliness and living alone are not overlapping concepts, but they are linked. Research showed that those without immediate kin are more likely to live alone than their peers with such kin in almost all countries [51,52], which creates an objective state of social isolation. This state is related to a lack of daily care and social support for older adults, causing them to tend to have poorer self-rated health and are more likely to be socioeconomically disadvantaged, which could lead to subjective feelings of loneliness.

As the commonly recognized important social determinants of health, the social indicators were also verified by this study as the relevant factors for the level of loneliness in the Hakka elderly. Specifically, we found that those who were still engaged in labor work and those with worse self-rated financial status and lower education levels obtained a higher score of ULS-8, which reveals a “disadvantage accumulation” phenomenon. In general, older persons who were still engaged in labor work may indicate a poorer family economic situation, which requires the retired elderly to return to the labor market to support the family. While economical restrictions not only caused material problems but also affected the interpersonal relationship and evoked feelings of loneliness [53]. People with higher economic levels usually have better living and working conditions; they have access to strong social support and high-quality resources. Moreover, higher educated older adults generally have better-tackling abilities and more social resources to enrich their life, which help them experience less loneliness. A surprising finding in this study is that the type of medical insurance was significantly associated with loneliness among the Hakka elderly, which seems to be strangeness. However, participants with different types of medical insurance tended to have widely varying occupations. Especially in Ninghua, where older adult predominantly has an agricultural hukou, those who possessed the Urban Employees Basic Medical Insurance (UEBMI) were mostly government employees, while those who hold the Urban and Rural Residents Basic Medical Insurance (URRBMI) were mainly farmers. There is also a huge gap between the two types of medical insurance in the level of health service benefits. Thus, the type of medical insurance reflects the socioeconomic status of the participants, and it may be an indirect predictor of loneliness. As one of the distinguishing indicators of identity, it also reminds us of the need to focus on vulnerable populations such as farmers.

## 5. Conclusion

To the best of our knowledge, this is the first study targeting the Hakka elderly to reveal their loneliness status and related factors. The present study provides an overall understanding of the loneliness among the Hakka elderly in Fujian. The results of this study showed that the loneliness of the Hakka elderly was moderate and slightly lower than at the national level. Sex, health status, regular exercise, leisure activities, healthy diet, smoking, marital status, residence, living arrangement, survival of parents, working status, financial status, education level, and type of medical insurance are identified to be the most significant predictors to affect the loneliness status of the Hakka elderly. The present study also obtained baseline information useful to the local government in their attempts to reduce the loneliness level of the Hakka elderly. Our findings suggest that relevant health interventions, programs, and support initiatives should be implemented in a targeted manner, focusing on susceptible populations. More specifically, the joint efforts (humanistic care and social support) of families, government organizations, and community members should give priority to vulnerable groups who are perceived to be at a higher level of loneliness among the Hakka elderly.

## 6. Limitations

There are several limitations of this study that should be noted. Firstly, the study is based on a cross-sectional survey; thus, the causal relationship between the variables and loneliness cannot be ascertained. Secondly, considering the fact that the education level of the Hakka elderly in the survey area is generally low and the communication barriers caused by the local dialect, some of the surveys were completed with the assistance of the elderly family caregivers. So there may be some discrepancy in the understanding of the participants and their family caregivers, which could lead to a certain bias. Thirdly, the Hakka people are widely distributed in Guangdong and Jiangxi in China and other southeast Asian countries such as Thailand, Malaysia, and Singapore, and the Hakka elderly in this study were only from Fujian, China. Therefore, the results may not necessarily be generalizable to the Hakka elderly in other regions. Lastly, nonresponse bias was not assessed, as only those agreeing to participate were included in the study analyses.

## Figures and Tables

**Figure 1:** Theoretical framework of the study.

**Table 1:** Demographic characteristics and ULS-8 scores of the study sample.

Layers	Variables	Categories	*N* (%)	Mean ± SD	*t*/*F*	*P*
Individual indicators	Sex	Male	613 (48.57)	15.23 ± 6.48	−5.363	<0.001
		Female	649 (51.43)	17.26 ± 6.95		
	Age	60–64	356 (28.21)	16.19 ± 6.63	0.295	0.881
		65–69	248 (19.65)	15.96 ± 6.54		
		70–74	227 (17.99)	16.43 ± 7.69		
		75–79	204 (16.16)	16.28 ± 7.10		
		≥80	227 (17.99)	16.59 ± 6.13		
	Self-rated health status	Very good/good	374 (29.64)	12.28 ± 4.08	196.229	<0.001
		General	711 (56.34)	16.73 ± 6.69		
		Very poor/poor	177 (14.03)	22.89 ± 6.07		
	Number of NCDs	0	599 (47.46)	14.65 ± 5.94	55.497	<0.001
		1	388 (30.74)	16.38 ± 6.74		
		≥2	275 (21.79)	19.65 ± 7.37		

Behavioral indicators	Regular exercise	No	638 (50.55)	20.73 ± 6.06	31.652	<0.001
		Yes	624 (49.45)	11.71 ± 3.85		
	Leisure activities	No	498 (39.46)	21.25 ± 5.68	25.691	<0.001
		Yes	764 (60.54)	13.03 ± 5.36		
	Healthy diet	No	586 (46.43)	19.24 ± 6.84	15.559	<0.001
		Yes	676 (53.57)	13.70 ± 5.61		
	Smoking	Yes	282 (22.35)	19.50 ± 6.37	9.570	<0.001
		No	980 (77.65)	15.34 ± 6.64		
	Drinking	Yes	553 (43.82)	16.09 ± 6.83	-0.832	0.405
		No	709 (56.18)	16.41 ± 6.78		

Interpersonal indicators	Marital status	Married/cohabitation	843 (66.80)	14.33 ± 6.03	125.117	<0.001
		Widowed	291 (23.06)	19.89 ± 6.63		
		Others	128 (10.14)	20.84 ± 6.47		
	Current residence	Rural	478 (37.88)	21.61 ± 5.67	558.301	<0.001
		Suburban	274 (21.71)	16.61 ± 6.38		
		Urban	510 (40.41)	11.08 ± 2.94		
	Living arrangement	Living alone	104 (8.24)	22.68 ± 5.86	80.191	<0.001
		Living with spouse only	400 (31.70)	14.46 ± 6.19		
		Living with children	435 (34.47)	13.88 ± 5.50		
		Mixed habitation	235 (18.62)	19.90 ± 6.89		
		Others	88 (6.97)	19.07 ± 6.24		
	Survival of parents	Both died	741 (58.72)	17.54 ± 6.84	8.228	<0.001
		Father or/and mother alive	521 (41.28)	14.47 ± 6.32		

Social indicators	Working status	No	865 (68.54)	14.89 ± 6.34	−10.918	<0.001
		Still engaged in labor work	397 (31.46)	19.29 ± 6.80		
	Self-rated financial status	Very poor/poor	268 (21.24)	22.24 ± 5.18	253.870	<0.001
		General	761 (60.30)	15.86 ± 6.46		
		Very good/good	233 (18.46)	10.76 ± 3.40		
	Education level	Illiterate	674 (53.41)	20.02 ± 6.47	224.965	<0.001
		Literacy class/home school	192 (15.21)	12.36 ± 4.39		
		Primary school	192 (15.21)	11.82 ± 3.94		
		Junior high school and above	204 (16.16)	11.76 ± 3.90		
	Medical insurance	URRBMI	995 (78.84)	17.64 ± 6.76	111.484	<0.001
		UEBMI	165 (13.07)	11.03 ± 3.31		
		Uninsured/unknown	102 (8.08)	11.44 ± 4.78		

**Table 2:** Hierarchical linear regression analysis on the loneliness score of the Hakka elderly.

Layers	Variables	Categories	Model 1		Model 2		Model 3		Model 4	
			*β*	*P*	*β*	*P*	*β*	*P*	*β*	*P*
Individual indicators	Sex (ref = male)	Female	1.577	<0.001	1.403	<0.001	0.843	0.001	0.631	0.012
	Self-rated health status (ref = very good/good)	General	4.093	<0.001	1.851	<0.001	1.184	<0.001	0.819	0.004
		Very poor/poor	9.375	<0.001	4.524	<0.001	2.977	<0.001	2.457	<0.001
	Number of NCDs (ref = 0)	1	0.987	0.010	0.676	0.025	0.520	0.050	0.476	0.067
		≥2	2.600	<0.001	1.167	0.001	1.389	<0.001	1.340	<0.001

Behavioral indicators	Regular exercise (ref = no)	Yes			–4.930	<0.001	–2.837	<0.001	–2.494	<0.001
	Leisure activities (ref = no)	Yes			–2.520	<0.001	–2.006	<0.001	–1.937	<0.001
	Healthy diet (ref = no)	Yes			–2.067	<0.001	–1.365	<0.001	–1.270	<0.001
	Smoking (ref = Yes)	No			–0.304	0.391	0.345	0.272	0.348	0.261

Interpersonal indicators	Marital status (ref = married/cohabitation)	Widowed					0.713	0.042	0.944	0.008
		Others					0.651	0.136	0.605	0.163
	Current residence (ref = urban)	Rural					6.167	<0.001	4.863	<0.001
		Suburban					2.700	<0.001	2.027	<0.001
	Living arrangement (ref = living with children)	Living alone					1.096	0.036	0.322	0.537
		Living with spouse only					0.289	0.317	0.327	0.262
		Mixed habitation					0.970	0.008	0.518	0.157
		Others					0.405	0.411	–0.275	0.576
	Survival of parents (ref = father or/and mother alive)	Both died					0.860	0.001	0.886	0.001

Social indicators	Working status (ref = no)	Still engaged in labor work							1.128	<0.001
	Self-rated financial status (ref = very poor/poor)	General							–1.376	<0.001
		Very good/good							–2.024	<0.001
	Education level (ref = illiterate)	Literacy class/home school							–1.527	<0.001
		Primary school							–1.370	0.002
		Junior high school and above							–2.105	<0.001
	Medical insurance (ref = URRBMI)	UEBMI							0.852	0.030
		Uninsured/Unknown							0.672	0.173
	***F***		<0.001		<0.001		<0.001		<0.001	
	***R*** ^***2***^		0.270		0.550		0.662		0.680	

## Data Availability

The data sets generated and/or analyzed during the current study are available from the corresponding author upon reasonable request.
